RETRACTED

# Rice Drought Damage Assessment Using AMSR-E Data Inversion of Surface Temperature

**DOI:** 10.1155/2022/4117481

**Published:** 2022-05-17

**Authors:** Ying Wang, Jianping Zhang, Guochun Li

**Affiliations:** ^1^Chongqing Institute of Meteorological Sciences, Chongqing 401147, China; ^2^Jiangjin Modern Agrometeorological Experiment Station of Chongqing, Jiangjin, Chongqing 402260, China; ^3^Jiangjin Meteorologica Administration, Jiangjin, Chongqing 402260, China

## Abstract

The extreme drought events caused by global warming have become one of the major issues of general concern all over the world. It is estimated that over the past 50 years, the average annual drought-affected area has reached more than 200,000 km^2^, resulting in a global economic loss of US$6-8 billion, far exceeding other meteorological disasters. Therefore, conducting real-time and effective drought monitoring research is of great significance for issues such as climate change, drought defense, water resources management, and protection in various regions. Rice is the largest food crop in China and plays a pivotal role in food production. Drought is often regarded as one of the most important stress factors. Scientific, accurate, and timely assessment of the impact of drought on rice yield is essential for improving crop drought resistance and ensuring food production. In this study, based on the meteorological data, rice growth period and yield of the main rice planting areas in Chongqing Yangtze River Basin, and based on the drought index of passive microwave remote sensing observation data (AMSR-E), a statistical model of rice meteorological yield and drought index under the influence of drought is established. A rice drought disaster assessment is carried out. The results of the disaster assessment indicate that under the influence of drought, the rice yield reduction rate of representative sites in Chongqing Yangtze River Basin is between 3% and 10%.

## 1. Introduction

As a kind of agricultural disaster, dry early morning has a significant impact on the society and economy, especially for rice production. Rice is the main grain type and food crop in China. It is the main food source for the world's Chinese population and is also an important economic source for China's 500 million farmers. Especially in the southern region, which accounts for 40% of China's land area and 60% of the country's population, it provides 90% of the country's rice output. Although the proportion of rice production in the southern region has declined in recent years, the importance of rice in the southern region has not changed [1–3].

Rice production is a kind of agricultural production, which is greatly restricted by natural conditions, especially by precipitation and irrigation conditions. Due to the great differences in geography and climate among different regions of China, the rice-producing regions in China can be divided into two rice regions, south and north, with the Qinling, Huaihe and Yangtze River lines as the boundaries. The area to the south is the rice area in southern China [4]. The southern region of China is generally rich in precipitation, but because of its vast territory and complex geographical environment, the natural conditions (such as heat and rainfall), and economic and social conditions of the provinces and cities in the southern region are not the same. Production conditions are also different. Among them, drought is one of the important factors affecting rice production in southern China. For example, in 2003, Hunan, Jiangxi, Zhejiang, Fujian, and other provinces in southern China experienced the worst drought since 1971. Since rice is the most water-intensive food crop among crops grown in southern China, it was also affected the most during this drought, and the government and farmers paid a heavy price for it [5–7].

RETRACTED

Drought is a water shortage caused by the imbalance of water supply and demand. It has the characteristics of high frequency, long duration, and wide range of influence. Drought index is the basis for studying arid climate, and it is also a key link to measure the degree of drought. At present, there are mainly two types of drought monitoring indicators widely used at home and abroad: one is mainly based on the ground climate data observed at a single point to construct a drought index, and the research on these traditional drought indices is mainly based on deterministic forecasts [8]. It is very easy to be affected by the initial conditions, resulting in inaccurate monitoring results, which will be difficult to effectively reflect the drought situation; the other is the drought monitoring index based on modern satellite remote sensing information, mainly using multi-temporal and multi-spectral, multi-angle remote sensing data through various methods to construct drought index to qualitatively or quantitatively evaluate soil moisture distribution from different aspects. The construction of drought index based on remote sensing information for monitoring has the characteristics of wide range and high spatial resolution, which is of great significance for the monitoring of drought in the human range [9–11].

Soil moisture is an important factor in determining the temporal and spatial dynamic changes of agricultural drought. Soil moisture remote sensing inversion technology overcomes the shortcomings of traditional soil moisture measurement methods and is widely used in agricultural drought monitoring. Both optical remote sensing and microwave remote sensing can successfully detect soil moisture and monitor agricultural drought. Microwave remote sensing is based on the contrast between the dielectric constants of dry soil and water and is considered to be the most suitable monitoring method for soil moisture due to its working characteristics of all-day, all-weather, and certain penetration of soil and vegetation. Active microwave remote sensing has high spatial resolution, but is more susceptible to soil roughness and crops, and is suitable for small-scale soil moisture inversion [11, 12]. Passive microwave remote sensing has a short revisit period and is relatively less affected by roughness and terrain, but the spatial resolution of the images is relatively low, which is suitable for large-scale agricultural drought monitoring.

RETRACTED

Compared with infrared and visible light, passive microwave remote sensing has the advantages of long wavelength and strong penetrating ability. Compared with active microwave radar, passive microwave radiometer has the advantages of large monitoring area, short period, less influence by roughness, and less impact on soil moisture. It is more sensitive and the algorithm is more mature. Qiu Yubao et al. used the global surface soil moisture and rainfall rate data retrieved by passive microwave radiometer AMSR-E as the research object, analyzed the impact of precipitation on soil moisture retrieval and its temporal and spatial correlation characteristics, and analyzed the weak correlation between retrieval parameters. The reasons for the emergence were investigated. Alexander et al. studied the influence of soil surface disequilibrium on the use of passive microwave remote sensing to retrieve soil moisture at different scales (l–4 km) and considered the noise and additional information of the sensor, the brightness of the simulated soil surface conditions [13–15]. The temperature has also been comprehensively studied, and the soil moisture inversion is obtained through the simulation of multi-angle observations by the superposition method of brightness temperature. The uncertainty of soil moisture inversion is mainly caused by the pixel uncertainty of the surface data due to the noise of the sensor. Meanwhile, different spatial scales are studied.

This study takes Chongqing Yangtze River Basin as the research object, uses AMSR-E multi-channel microwave remote sensing data to construct a drought index, establishes a statistical model of rice meteorological yield and drought index under the influence of drought, and conducts rice drought disaster assessment [16, 17].

RETRACTED

## 2. Methods and Theory

### 2.1. Research Object

Chongqing is located in Southwest China and the upper reaches of the Yangtze River. It crosses the transition zone between the Qinghai Tibet Plateau and the plains in the middle and lower reaches of the Yangtze River between 105°11′∼110°11′ east longitude and 28°10′∼32°13′ north latitude. The main rivers in Chongqing include the Yangtze River, Jialing River, Wujiang River, Fujiang River, Qijiang River, Daning River, Apeng River, and Youshui River. The main stream of the Yangtze River crosses the whole territory from west to east, with a flow of 665 kilometers. Chongqing has a subtropicatechniq=l monsoon humid climate, with an annual average temperature of 16∼18°C, the average temperature in the hottest month of 26∼29°C and the average temperature in the coldest month of 4∼8°C. The annual average precipitation is abundant, with most areas ranging from 1000 mm to 1350 mm. The precipitation is mostly concentrated from May to September, accounting for about 70% of the total precipitation of the whole year. Chongqing has a cultivated land area of 1622000 hectares, with a high degree of agricultural cultivated land development and comprehensive development of agriculture, forestry, animal husbandry, and sideline fisheries. It is an important main grain producing area in China. Among them, the main grain crops include rice, corn, wheat, and sweet potato, especially rice.

### 2.2. Research Data Sources

The data used by Muwen includes the AMSR-E Level-3 data of each month in Chongqing Yangtze River Basin for 5 years from 2014 to 2019, from the National Snow and Ice Center (NSIDC) in the United States and from all meteorological observation stations in Chongqing Yangtze River Basin from 2010 to 2020 The daily precipitation data and the daily soil moisture data of all soil moisture monitoring stations in Chongqing Yangtze River Basin from 2010 to 2020 are obtained from the China Meteorological Administration.

### 2.3. AMSR-E Data Presentation

Advanced Microwave Scanning Radiometer AMSR-E (The Advanced Scanning Radiometer for EOS) is an improved design based on the AMSR sensor and was carried on the Aqua satellite of NASA's Earth Observing System (EOS) . AMSR-E is a full-energy passive microwave radiometer with cone scanning. The sensor can observe the range of 89.24N-89.24S. AMSR-E observes the Earth every day from 0 to 8 times, and at the same time every day, there will be some gaps between the swept bands. The AMSR-E data used in this study includes the brightness temperature values of 12 channels, the quality evaluation of the data, and the inversion value of the ground soil moisture. At the same time, the daily data includes orbital ascending and descending orbit data. The main difference between them is that the scanning direction of the sensor is different. The ascending orbit data is scanned from the South Pole to the North Pole, and the descending orbit data is scanned from the North Pole to the South Pole. The spatial resolution of the Level-3 terrestrial product (AELand3) used in this study has been resampled and unified to 25 km.

RETRACTED

### 2.4. Drought Index

When studying the surface vegetation, it is considered that due to photosynthesis, the absorption of light by plant chlorophyll is the reduction of redlight energy reflected by the growth of plants. At the same time, plants absorb little radiation in the infrared band. The reflection is in the infrared. Based on the principle that the energy of the plant increases with the growth of the plant, the vegetation index is constructed by means of the harmonic product quotient of the infrared band and the near-infrared band, and the polarization ratio. Therefore, according to this idea, this study uses the sum-difference quotient and other methods to construct the drought index for the 10 bands under the horizontal and vertical polarization modes of AMSR-E.

The brightness temperature Tb observed by AMSR-E is related to the ground reflectance *ε* and is expressed as

(1) $$\begin{array}{c} T_{b}=\varepsilon T_{s}. \end{array}$$

Among them, *T*_*b*_ is the surface brightness temperature value received by the satellite, which is related to soil properties, vegetation conditions, and ground roughness, etc., and the influence of soil moisture plays a major role; *T*_*s*_ is the surface temperature. At the same temperature, the microwave radiometer that received surface brightness temperature is related to *ε*, while *ε* is closely related to soil moisture content. *ε* varies from 0.95 to 0.6 from dry soil to water saturated soil. Therefore, the ratio of the information of different bands can be used to try to establish the drought index. The AMSR-E data used in this study lacks data in the 23.8 GHz band, and the selected drought index is TBv06.9/TBv36.5.

### 2.5. Rice Yield Assessment

The research object of this study is single-cropping rice. The data of rice growth period from agro-meteorological observation stations is collected and analyzed, and the time of transplanting, booting, flowering, and maturity in each rice planting area is obtained by combining with the actual survey data in the field. The rice transplanting area in Chongqing Yangtze River Basin is mid-June, the booting period is mid-August, the flowering period is early September, and the maturity period is mid-October.

RETRACTED

The statistical model of drought index and meteorological yield from transplanting to booting stage, booting to flowering stage, flowering to maturity stage can be expressed as

(2) $$\begin{array}{c} Y_{i}=A\times D_{1}+B\times D_{2}+C\times D_{3}+D. \end{array}$$

*Y*_*i*_ is the meteorological yield (kg/hm2); *D*_1_ is the drought index after standardization from transplanting to booting stage; *D*_2_ is the drought index after standardization from booting to flowering stage; *D*_3_ is the drought index after standardization from flowering to maturity; *A*, *B*, *C* is the coefficient; and *D* is a constant.

The reduction percentage of the actual rice yield after drought and the normal predicted yield without drought is given in the formula

(3) $$\begin{array}{c} Y_{d}=\frac{\left(Y_{P}-Y\right)}{Y_{P}}. \end{array}$$

In the formula: *Y*_*d*_ is the yield reduction rate; *Y*_*P*_ is the normal predicted yield without drought (the standardized drought index for each growth stage in equation (3) is taken as 0); and *Y* is the historical statistical yield.

## 3. Results and Discussion

### 3.1. AMSR-E Drought Index Verification

In this summary, based on the analysis of the actual meteorological conditions in Chongqing Yangtze River Basin from 2014 to 2019, and the distribution characteristics of stations in Chongqing Yangtze River Basin, this study selects a certain station in Chongqing Yangtze River Basin to study the correlation between drought index and drought in time series.

From Figure 1, it can be found that the site drought index is basically positively correlated with the measured soil moisture content. From the standard table of drought grade classification of soil relative humidity (Ms), it can be found that different degrees of drought occurred at site 1 during the test period, and the corresponding drought index reaches a large value, or a maximum value appeared immediately after an upward trend. It can be inferred that when the MPDI index is greater than 0.02, drought may occur in the region.

From the time-series graph of the station, it can be found that the drought index calculated from the AMSR-E brightness temperature data is similar to the change trend of the measured soil moisture, so the index is more suitable for drought monitoring in Chongqing Yangtze River Basin. However, it is predicted time is delayed, and the length of its delay needs to be considered in practical applications.

It can be known from Figure 2 that the site drought index and rainfall basically have a negative correlation trend; the brightness temperature data of the vertical polarization of AMSR-E is larger than that of the horizontal polarization, which is inconsistent with the general theory. Vegetation grows better in the rainy season, which affects the AMSR-E sensor to receive surface radiation, and the vegetation layer affects the sensitivity of the brightness temperature measured by the radiometer to the monitoring of soil moisture.

RETRACTED

The drought index can reflect the area and degree of drought due to lack of precipitation to a large extent, that is to say, the established ratio drought index can indicate drought to a certain extent. The drought index selected in this study can better reflect the drought caused by the sparse precipitation. Compared with the anomalous vegetation index and conditional vegetation index methods, the microwave method does not need to rely on the surface vegetation and has a high repeated observation rate and is real time. Due to the lower resolution of AMSR-E, the drought index is suitable for larger scale studies.

Due to the difference in solar radiation in each season, the difference in surface temperature causes the difference in surface radiance rate, so the range of dividing the drought index in each season is also different. Another important issue with the ratio drought index is the conversion between the calculated index and true soil moisture. The current research mainly uses the measured soil moisture data for regression, but the regression correlation coefficient is not high and the reliability is poor. Moreover, this method has the problem that the feature space indices of different time and different regions cannot be compared and analyzed. Precipitation and soil moisture are two very important parameters in meteorology, climate, hydrology, and ecological environment, and they are also the most active parts of the global water and energy cycle, and they are also important factors in the occurrence of drought. In the past, traditional drought monitoring methods relying on factors such as precipitation and soil moisture were mainly used, but these factors were few in measurement points, which made it difficult to achieve large-scale, real-time, and dynamic drought monitoring; the modern remote sensing inversion technology currently used is sufficient. Overcoming the shortcomings of traditional soil moisture monitoring methods, it has gradually been widely used in agricultural drought monitoring. Microwave remote sensing is based on the contrast between the dielectric constants of dry soil and water. It has the characteristics of all-day and all-weather monitoring, and has a certain penetrability to soil and vegetation. It is considered to be the most suitable monitoring method for soil moisture. Active microwave remote sensing is relatively easy to be affected by soil roughness and crops, and the amount of data is large and the data processing is complex, so it is suitable for small-scale inversion; passive microwave remote sensing has a short revisit period and is relatively less affected by roughness and terrain. It has the advantages of large-scale, macroscopic, and dynamic monitoring, but the spatial resolution of its images is relatively low, which is suitable for large-scale drought monitoring.

RETRACTED

### 3.2. Decadal Variation of Drought Index in Each Growth Period

#### 3.2.1. Transplant to Booting Stage

From 2014 to 2019, the change trend of drought index from transplanting to booting stage in the six major rice planting areas in Chongqing Yangtze River Basin shows that the average drought index of Fengdu County and Dianjiang County is much higher than that of other areas, 1.75 and 0.95, respectively, followed by Zhong County, Chengkou County, Yunyang County, and Fengjie County which are 0.53, 0.45, 0.37, and 0.26, respectively. The drought index showed a fluctuating trend.

#### 3.2.2. Booting to Flowering Stage

The variation trend of drought index from booting to flowering stage in six major rice planting areas in Chongqing Yangtze River Basin from 2014 to 2019 shows that the areas with severe drought from booting to flowering period were mainly Chengkou County, with an average drought index of 2.71; Dianjiang County and Fengdu County followed, with 2.05, 1.73, respectively; Yunyang County, Fengjie County, and Zhong County had the lowest, with 0.69, 0.55, and 0.41, respectively.

#### 3.2.3. Flowering to Maturity

From 2014 to 2019, the variation trend of drought index from flowering to maturity in the six major rice planting areas in Chongqing Yangtze River Basin shows that the areas with severe drought from flowering to maturity are mainly Dianjiang County and Chengkou County, with the mean values of the drought index being 1.05 and 0.78, respectively, followed by Fengdu County, Fengjie County, Yunyang County, and Zhong County is the lowest.

The above 6 representative statistical models of rice trend yield are from 2014 to 2019 at the site. The trend yield is obtained by separating the actual yield data using orthogonal polynomials. The statistical models of the rice trend yield of representative sites in different rice planting areas are as follows:

(4) $$\begin{array}{c} \text{Chengkou County}Y=-0.05t^{3}+0.689t^{2}+70.234t+4589.9\;{\text{R}}^{2}=0.61,\\ \text{Fengdu County}Y=-0.268t^{3}+1.936t^{2}+20.569t+5196.5\;{\text{R}}^{2}=0.66,\\ \text{Dianjiang County}Y=0.459t^{3}-10.265t^{2}+205.673t+5235.1\;{\text{R}}^{2}=0.79,\\ \text{Zhoung County}Y=-0.698t^{3}+2.615t^{2}+333.216t+4498.6\;{\text{R}}^{2}=0.71,\\ \text{Yunyang County}Y=1.039t^{3}-38.296t^{2}+959.632t+6103.9\;{\text{R}}^{2}=0.79,\\ \text{Fengjie County}Y=0.513t^{3}-21.326t^{2}+323.59t+5153.6\;{\text{R}}^{2}=0.66. \end{array}$$

In drought years, the statistical model established to analyze the relationship between the drought index from transplanting to booting stage, booting to flowering stage, and flowering to maturity stage and meteorological yield is as follows:

(5) $$\begin{array}{c} \text{Chengkou County}Y=70.35-365.22D_{1}+202.63D_{2}-99.186D_{0},\\ \text{Fengdu County}Y=145.63-504.88D_{1}+101.693D_{2}-78.26D_{0},\\ \text{Dianjiang County}Y=165.43-156.93D_{1}+77.82D_{2}-115.88D_{0},\\ \text{Zhoung County}Y=169.42-226.55D_{1}+89.63D_{2}-102.32D_{0},\\ \text{Yunyang County}Y=248.69-65.77D_{1}+243.62D_{2}-108.54D_{0},\\ \text{Fengjie County}YY=59.52-196.52D_{1}+245.36D_{2}-177.81D_{0}. \end{array}$$

RETRACTED

### 3.3. Rice Drought Disaster Assessment

The comparative analysis represents the difference between the measured rice yield and the simulated yield in the dry years of the site. Figures 3 and 4 show that the absolute value of the relative error between the two is less than 3.5%, which not only shows that the established model can objectively reflect the drought of rice in different growth periods. The impact on yield can also better assess the loss of rice yield under the influence of drought. At the same time, according to the rice drought disaster assessment model, the measured yield after drought and the normal predicted yield after drought in representative sites in each planting area are analyzed. It can be seen from Figure 5 that under the influence of drought, the rice yield reduction rate of each representative site is 4–10%.

## 4. Conclusion

1. This study analyzes the time-series relationship between the drought index and the daily precipitation index at the measured stations in the study area, and obtains the time-series diagram of the drought index and the daily precipitation and the standardized precipitation index at the measured stations. The drought index selected in this study can fully reflect the drought situation of the site and is suitable for drought research in Chongqing Yangtze River Basin.
2. Drought disasters have been one of the main natural disasters in Southwest China since ancient times, and also one of the main agro-meteorological disasters that restrict the sustainable and stable development of agriculture, and have a great impact on the formation of rice yields. In this study, the drought index TBv06.9/TBv36.5 in the MSR-E data is selected based on the comprehensive consideration of crops, atmosphere, and soil in Sichuan rice area, and the drought index is verified by using the actual disaster data, and the effect is good.
3. In this study, six representative sites are selected in Chongqing Yangtze River Basin rice planting area for analysis, but the topography in the same area is complex. There are differences in meteorological factors and crop growth periods, and there are certain differences in the evaluation within the region. Due to the impact of other disasters such as high temperature, floods, rain, diseases and insect pests, the reasons for the loss of rice yield may include other meteorological disasters, and how to completely separate the impact of drought on crop yield needs to be further studied. In addition, the objectivity and accuracy of the data obtained also affect the research results. Today, the accuracy of agricultural meteorological observation data in various places is not high, coupled with insufficient data, resulting in great uncertainty in the results. Of course, with the improvement of observation data and the improvement of research indicators, the results will be more and more accurate.

RETRACTED

## Figures and Tables

**Figure 1:** Comparison of time series between drought index and measured soil moisture content.

**Figure 2:** Comparison of drought index and rainfall time series.

**Figure 3:** Comparison of the product of the real value and predicted value in 2008.

**Figure 4:** Comparison of the product of the real value and predicted value in 2018.

**Figure 5:** Rice disaster assessment in Chongqing Yangtze River Basin in 2018.

## Data Availability

The figures data used to support the findings of this study are included in the article.

## References

[1] Kang H., Sridhar V., Mainuddin M., Trung L. D. (2021). Future rice farming threatened by drought in the Lower Mekong Basin. *Scientific Reports*.

[2] Van Nguyen N., Ferrero A. (2006). Meeting the challenges of global rice production. *Paddy and Water Environment*.

[3] Peng S., Tang Q., Zou Y. (2009). Current status and challenges of rice production in China. *Plant Production Science*.

[4] Muthayya S., Sugimoto J. D., Montgomery S., Maberly G. F. (2014). An overview of global rice production, supply, trade, and consumption. *Annals of the New York Academy of Sciences*.

[5] Bouman B. A. M. (2001). Water-efficient management strategies in rice production. *International Rice Research Notes*.

[6] Panuju D. R., Mizuno K., Trisasongko B. H. (2013). The dynamics of rice production in Indonesia 1961-2009. *Journal of the Saudi Society of Agricultural Sciences*.

[7] Simatupang P., Peter Timmer C. (2008). Indonesian rice production: policies and realities. *Bulletin of Indonesian Economic Studies*.

RETRACTED

[8] Tuong T. P. (2000). Productive water use in rice production. *Journal of Crop Production*.

[9] Hu L., Zhang J., Ren W. (2016). Can the co-cultivation of rice and fish help sustain rice production?. *Scientific Reports*.

[10] Rehman H.-u., Aziz T., Farooq M., Wakeel A., Rengel Z. (2012). Zinc nutrition in rice production systems: a review. *Plant and Soil*.

[11] Du J., Kimball J. S., Velicogna I. (2019). Multicomponent satellite assessment of drought severity in the contiguous United States from 2002 to 2017 using AMSR‐E and AMSR2. *Water Resources Research*.

[12] Zhang H., Wang S., Liu K. (2022). Downscaling of AMSR-E soil moisture over north China using random forest regression. *ISPRS International Journal of Geo-Information*.

[13] Zhu Q., Luo Y., Xu Y.-P., Tian Y., Yang T. (2019). Satellite soil moisture for agricultural drought monitoring: assessment of SMAP-derived soil water deficit index in Xiang River Basin, China. *Remote Sensing*.

[14] Bai J., Cui Q., Chen D. (2018). Assessment of the SMAP-derived soil water deficit index (SWDI-SMAP) as an agricultural drought index in China. *Remote Sensing*.

[15] Yang S., Zhang D., Sun L., Wang Y., Gao Y. (2020). Assessing drought conditions in cloudy regions using reconstructed land surface temperature. *Journal of Meteorological Research*.

[16] Sun X., Wang M., Li G., Wang Y. (2020). Regional-scale drought monitor using synthesized index based on remote sensing in northeast China. *Open Geosciences*.

[17] Yang J., Zhang P., Lu N., Yang Z., Shi J., Dong C. (2012). Improvements on global meteorological observations from the current Fengyun 3 satellites and beyond. *International Journal of Digital Earth*.

